# Glaucocalyxin A Attenuates IL-1*β*-Induced Inflammatory Response and Cartilage Degradation in Osteoarthritis Chondrocytes via Inhibiting the Activation of NF-*κ*B Signaling Pathway

**DOI:** 10.1155/2022/6516246

**Published:** 2022-02-26

**Authors:** Weidong Zhu, Yi Zhang, Yueshan Li, Hao Wu

**Affiliations:** ^1^The Department of Orthopedics, The Second Affiliated Hospital of Xi'an Jiaotong University, Xi'an, 710004 Shaanxi Province, China; ^2^The Department of Ophthalmology, The Second Affiliated Hospital of Xi'an Jiaotong University, Xi'an, 710004 Shaanxi Province, China; ^3^The Department of Stomatology, The First Affiliated Hospital of Xi'an Jiaotong University, Xi'an, 710061 Shaanxi Province, China

## Abstract

Glaucocalyxin A (GLA) is a bioactive natural compound with anti-inflammatory activity. Herein, the role of GLA in osteoarthritis (OA) was evaluated. Our results demonstrated that the IL-1*β*-induced inducible nitric oxide synthase (iNOS) and cyclooygenase-2 (COX-2) expression, two enzymes resulting in the release of nitric oxide (NO) and PGE2, were also prevented by GLA in chondrocytes. Moreover, GLA suppressed inflammatory cytokines production in chondrocytes. In addition, the elevated expressions of MMPs and ADAMTSs and the degradation of aggrecan and collagen II were reversed by GLA in chondrocytes. Furthermore, GLA decreased p-p65 level and suppressed the nuclear p65 accumulation in the nucleus of chondrocytes. Collectively, we concluded that GLA attenuated inflammatory response in chondrocytes via NF-*κ*B pathway. These findings suggested that GLA might become an effective agent for OA treatment.

## 1. Introduction

Osteoarthritis (OA) is a frequent inflammation-related disease affecting individuals over 60 years of age [1]. OA is clinically presented with crepitus, joint pain, stiffness, tenderness, and limited movement [2]. Thus, OA patients commonly suffer with functional decline as well as loss of life quality, accompanied by heavy health care and society costs. Although osteoarthritis management consists of joint replacement for end-stage disease, the prevention and the treatment of early OA are still limited [1].

The identification of risk factors and understanding of the pathogenesis are central for selecting targets for OA therapy. It is evident for the role of chronic inflammation in the development of OA [3, 4]. Inflammation contributes to the evolution of joint tissue degradation and remodeling as well as joint pain [5]. A plethora of inflammatory mediators and signaling pathways are involved in the OA pathogenesis, which become potential biomarkers or therapeutic targets [6]. It is increasingly evident that interleukin-1*β*- (IL-1*β*-) mediated signaling pathways play central roles in OA pathology [7]. It is believed that components in the IL-1*β* signaling may be developed into novel drugs for OA.

Glaucocalyxin A (GLA), a bioactive natural compound, possesses important biological activities including anti-inflammatory activity [8–12]. Its chemical structure is shown in Figure 1(a). The administration of GLA reduces inflammation and mortality in lipopolysaccharide- (LPS-) induced septic-shock mouse model through regulating NLRP3 inflammasome activation [13]. Another study has proven that the LPS-stimulated increased production of proinflammatory cytokines in microglia is inhibited by GLA treatment [14]. Moreover, treatment with GLA reduces the inflammatory response in hydrogen peroxide- (H_2_O_2_-)induced smooth muscle cells [15].

Herein, we examined the potential role of GLA in OA. Evidence has been building that the inflammatory process in chondrocytes plays crucial role in the joint injury. Thus, IL-1*β*-induced chondrocytes are generally applied for in vitro model of OA [7]. Herein, we examined the effect of GLA on inflammation in chondrocytes.

## 2. Materials and Methods

### 2.1. Cell Culture and Treatment

Articular cartilage samples were obtained from articular joints of OA patients undergoing total knee replacement surgery. Primary human OA chondrocytes were then harvested from these clinical samples as previously described [16]. The resulting cells were centrifuged and cultured for our following study.

The experiments were divided into five groups: control, IL-1*β*, IL − 1*β* + GLA (5 *μ*M), IL − 1*β* + GLA (10 *μ*M), and IL − 1*β* + GLA (20 *μ*M).

### 2.2. Cell Viability Assay

We performed cell viability assay using CCK-8 kit (Promega Corp, Madison, WI). After the treatment with GLA (0, 5, 10, 20, and 40 *μ*M; Yuanye BioTech, Shanghai, China), the cells were treated with CCK-8 for 4 h. The OD value was measured at 450 nm.

### 2.3. Measurement of Nitric Oxide (NO)

Primary human OA chondrocytes were incubated with different concentrations of GLA (0, 5, 10, and 20 *μ*M) for 2 h and then stimulated with IL-1*β* (10 ng/ml) for 24 h. NO accumulation was measured using a commercial assay kit (Dojindo Laboratories, Kumaoto, Japan). The absorbance at 550 nm was measured and calculated for NO accumulation.

### 2.4. qRT-PCR

The total RNA from human OA chondrocytes was used for cDNA synthesis with cDNA Reverse Transcription Kit. The obtained cDNA was used for qRT-PCR. The primer sequences used are listed as follows: inducible nitric oxide synthase (iNOS), 5′-GAA ACT TCT CAG CCA CCT TGG-3′, and 5′-CCG TGG GGC TTG TAG TTG AC-3′; cyclooygenase-2 (COX-2), 5′-GGT GAA AAC TGT ACT ACG CCG A-3′, and 5′-ACT CCC TTG AAG TGG GTC AG-3′; TNF-*α*, 5′-CAT CTT CTC AAA ATT CGA GTG ACA A-3′, and 5′-TGG GAG TAG ACA AGG TAC AAC CC-3′; IL-6, 5′-AGA AAT CCC TCC TCG CCA AT-3′, and 5′-AAA TAG CGA ACG GCC CTC A-3′; IL-8, 5′-GCC CTC CTC CTG GTT TCA G-3′, and 5′-TGG CAC CGC AGC TCA TT-3′; matrix metalloproteinase (MMP)-3, 5′-TGA GGA CAC CAG CAT GAA CC-3′, and 5′-ACT TCG GGA TGC CAG GAA AG-3′; MMP-13, 5′-GCC ATT ACC AGT CTC CGA GG-3′, and 5′-TAC GGT TGG GAA GTT CTG GC-3′; A disintegrin-like and metalloproteinase with thrombospondin type I motifs (ADAMTS)-4, 5′-CAT CCT ACG CCG GAA GAG TC-3′, and 5′-AAG CGA AGC GCT TGT TTC TG-3′; ADAMTS-5, 5′-CCC AAA TAC GCA GGT GTC CT-3′, and 5′-ACA CAC GGA GTT GCT GTA GG-3′; aggrecan, 5′-AAG TGC TAT GCT GGC TGG TT-3′, and 5′-GGT CTG GTT GGG GTA GAG GT-3′; collagen II, 5′-CTC AAG TCG CTG AAC AAC CA-3′, and 5′-GTC TCC GCT CTT CCA CTC TG-3; and *β*-actin, 5′-ACT CTT CCA GCC TTC CTT CC-3′, and 5′-TGT TGG CGT ACA GGT CTT TG-3′.

### 2.5. Western Blot

Control and treated chondrocytes were lysed, followed by SDS-PAGE electrophoresis as previously described [13]. The primary antibodies used were listed: anti-iNOS, anti-COX-2, anti-*β*-actin, and HRP-conjugated secondary antibody from Santa Cruz Biotechnology, Santa Cruz, CA; and anti-ADAMTS-4, anti-ADAMTS-5, anti-aggrecan, anti-collagen II, anti-p65, anti-p-p65, anti-p-I*κ*B*α*, and anti-I*κ*B*α* from Abcam. Finally, the bands were visualized with the ECL reagent.

### 2.6. Elisa

The culture supernatants of chondrocytes were collected, centrifugated, and frozen at -80°C until assayed. Prostaglandin E2 (PGE2), TNF-*α*, IL-6, IL-8, and MMP-3 and MMP-13 contents were measured by ELISA (Boster Immunoleader, Pleasanton, CA).

### 2.7. Immunofluorescence Staining

After the completion of treatment, chondrocytes were fixed, permeabilized, and blocked for 1 h. Then, cells were probed with anti-p65 antibody (Abcam) overnight, followed by an incubation with ant-rabbit Alexa Fluor 546 secondary antibodies for 2 h. Cells were then mounted with DAPI and visualized by Olympus FV1000 confocal microscope (Olympus, Tokyo, Japan).

### 2.8. Statistical Analysis

Experimental data are presented as mean ± S.E.M. ANOVA was performed to show the difference between groups. *p* < 0.05 was considered as significant difference.

## 3. Results

### 3.1. Effect of GLA on OA Chondrocyte Viability

According to the results of Figure 1(b), GLA did not exhibit obvious cytotoxic effect on chondrocytes at the doses of 5, 10, and 20 *μ*M. Hence, these three concentrations were used for the next experiments.

### 3.2. Effect of GLA on NO and PGE2 Production

A rapid increase in the NO production was observed in IL-1*β*-induced chondrocytes, and this response was mitigated in the GLA-treated groups (Figure 2(a)). Besides, an acute increase in PGE2 content was noted in response to induction with IL-1*β*, while the GLA-treated chondrocytes showed significant mitigation in PGE2 content (Figure 2(b)).

### 3.3. Effect of GLA on iNOS and COX-2 Expression

IL-1*β* could increase the mRNA levels of iNOS and COX-2, these effects were reversed by GLA (Figures 3(a) and 3(b)). Chondrocytes in the IL-1*β*-treated group had significant higher protein levels of iNOS and COX-2, while GLA suppressed these proteins expression (Figure 3(c)).

### 3.4. Effect of GLA on Inflammatory Cytokine Production

QRT-PCR demonstrated that the mRNA levels of TNF-*α*, IL-6, and IL-8 were upregulated evidently in the IL-1*β*-stimulated group. However, in comparison with the IL-1*β* group, the mRNA levels were markedly decreased in the GLA-treated chondrocytes (Figures 4(a)–4(c)). Similarly, the contents of inflammatory factors were significantly induced by IL-1*β*, which were attenuated in the GLA-treated chondrocytes (Figures 4(d)–4(f)).

### 3.5. Effect of GLA on the Expression of MMPs

According to the results of qRT-PCR, chondrocytes in the IL-1*β*-stimulated group had increased mRNA levels of MMP-3 and MMP-13. While compared to the IL-1*β*-treated group, chondrocytes in the GLA-treated group had lower expressions of MMPs at mRNA level (Figures 5(a) and 5(b)). In addition, the results of ELISA assay indicated that GLA greatly inhibited the production of MMPs in chondrocytes (Figures 5(c) and 5(d)).

### 3.6. Effect of GLA on the Expression of ADAMTSs

Compared to the control group, the mRNA levels of ADAMTS-4 and ADAMTS-5 in the chondrocytes from the IL-1*β*-treated group were significantly increased, which were suppressed by GLA treatment (Figures 6(a) and 6(b). In addition, we observed that IL-1*β* greatly increased the protein levels of ADAMTS-4 and ADAMTS-5, which were downregulated after the pretreatment with GLA (Figure 6(c)).

### 3.7. Effect of GLA on the Expression of Aggrecan and Collagen II

IL-1*β* could decrease the mRNA expression levels of aggrecan and collagen II. However, GLA upregulated the mRNA expression levels of aggrecan and collagen II in OA chondrocytes (Figures 7(a) and 7(b)). Similarly, the western blot assay revealed comparable results in aggrecan and collagen II protein expression levels (Figure 7(c)).

### 3.8. Effect of GLA on the NF-*κ*B Pathway

The results from immunofluorescence indicated that IL-1*β* induced p65 nuclear accumulation, whereas the p65 accumulation was prevented by GLA (Figure 8(a)). The phosphorylation levels of p65 and I*κ*B*α* were increased in the IL-1*β*-treated chondrocytes, while I*κ*B*α* level was greatly decreased by IL-1*β* treatment. However, GLA prevented NF-*κ*B activation in the IL-1*β*-treated chondrocytes (Figures 8(b) and 8(c)).

## 4. Discussion

The recent work in OA-associated field has implicated inflammatory chemokines in OA pathogenesis. Interleukins are a big family of cytokines that comprises 11 members that shared similar gene structure [17]. IL-1*β* is involved in the pathology of OA [7]. IL-1*β* binds to the type I IL-1RI [18]. It was reported that increased levels of IL-1RI are detected in isolated chondrocytes. It is evident that during inflammatory processes, increased IL-1*β* increases IL-1RI expression. The extracellular domain of IL-1RI causes IL-1 receptor accessory protein recruitment, which is considered a coreceptor for IL-1*β* signal transduction [7]. Next, the signal transduction causes the activation of MAPK pathways and eventually results in various transcription factors activation, such as NF-*κ*B [7]. Collectively, IL-1*β* signaling is necessary for the development of OA and serves as a therapeutic target.

Here, we used IL-1*β* to induce an in vitro inflammatory OA model in chondrocytes, thereby exploring the anti-inflammatory effect of GLA exposed to IL-1*β* induction. IL-1*β* produces the production of proinflammatory cytokines, further induces iNOS expression, which results in NO accumulation [19]. Moreover, NO level is highly increased in OA chondrocytes as well as cartilage tissues [20]. NO inhibits the synthesis of proteoglycan and collagen and activates MMPs [21, 22]. Our results proved that GLA suppressed iNOS expression and NO release in chondrocytes. Like NO, PGE2, a predominant product of COX-2, is also increased during the progression of OA [19]. In human chondrocytes, the induction with IL-1*β* causes increased PGE2 release via regulating p38 MAPK pathway [23]. We also found that GLA suppressed the COX-2 expression and PGE2 release in IL-1*β*-induced chondrocytes.

In addition to acting as a key proinflammatory cytokine, IL-1*β* also contributes to the OA progression via mediating other events, such as inducing the expression of MMPs and ADAMTSs, which are cartilage-degrading enzymes [24–26]. IL-1*β* stimulates chondrocytes to release several types of MMPs, and these three proteases become a strategy to prevent OA [27, 28]. Moreover, the ADAMTS family of proteins, especially ADAMTS-4 and ADAMTS-5, is also important in cartilage degradation [29]. We found that the elevated expression of MMPs and aggrecan and collagen II degradation were reversed by GLA in chondrocytes.

The NF-*κ*B plays a crucial role in inflammation through modulating activation or repression of target gene expression [30]. Consequently, NF-*κ*B is essential in various inflammatory diseases including OA [31]. NF-*κ*B mediates critical inflammatory events by modulating chondrocytes, results in progressive extracellular matrix (ECM) damage [32]. The NF-*κ*B signaling was found to be regulated by IL-1*β* in OA chondrocytes [33]. Thus, we evaluated the role of GLA in NF-*κ*B pathway. NF-*κ*B is commonly presented in an inactive form in the cytoplasm associated with the inhibitory *κ*B proteins (I*κ*B) [34]. The I*κ*B*α* is an important mechanism for the activation and repression of NF-*κ*B [35]. We found that GLA decreased the levels of p-p65 and suppressed the p65 accumulation in nucleus, which indicated that GLA prevented NF-*κ*B pathway activation [36].

There existed several limitations in this study. A major limitation is that our results are based on the in vitro experiments. Future in vivo experiments are needed to verify the role of GLA in OA. Secondly, the exact molecular mechanisms by which GLA regulates NF-*κ*B pathway need to be further explored in the future study.

In light of this, we concluded that GLA attenuated the inflammatory response and cartilage degradation in chondrocytes via the regulation of NF-*κ*B. Thus, GLA might become an effective therapeutic agent for OA.

## Figures and Tables

**Figure 1:** Examination of cytotoxicity effect of GLA on human OA chondrocytes. (a) The chemical structure of GLA. (b) Primary human OA chondrocytes were prepared and incubated with different concentrations of GLA (0, 5, 10, 20, and 40 *μ*M) for 24 h. Subsequently, cells were processed to test the cell viability using CCK-8 assay. Experiments were performed at least in triplicate. ^∗^*p* < 0.05 versus the control group.

**Figure 2:** GLA inhibits the production of NO and PGE2 in IL-1*β*-stimulated OA chondrocytes. Primary human OA chondrocytes were incubated with different concentrations of GLA (0, 5, 10, and 20 *μ*M) for 2 h and then stimulated with IL-1*β* (10 ng/ml) for 24 h. (a) NO production was evaluated using the Griess reaction. (b) PGE2 content in culture supernatant was determined using ELISA. ^∗^*p* < 0.05 versus the control group; #*p* < 0.05 versus the IL-1*β* group.

**Figure 3:** GLA inhibits the expression of iNOS and COX-2 in IL-1*β*-stimulated OA chondrocytes. Primary human OA chondrocytes were incubated with different concentrations of GLA (0, 5, 10, and 20 *μ*M) for 2 h and then stimulated with IL-1*β* (10 ng/ml) for 24 h. (a and b) The mRNA levels of iNOS and COX-2 were evaluated using qRT-PCR. (c) The protein levels of iNOS and COX-2 were evaluated using western blot. ^∗^*p* < 0.05 versus the control group; #*p* < 0.05 versus the IL-1*β* group.

**Figure 4:** Modulation of TNF-*α*, IL-6, and IL-8 production by GLA in human OA chondrocytes. Primary human OA chondrocytes were incubated with different concentrations of GLA (0, 5, 10, and 20 *μ*M) for 2 h and then stimulated with IL-1*β* (10 ng/ml) for 24 h. (a–c) The mRNA levels of TNF-*α*, IL-6, and IL-8 were evaluated using qRT-PCR. (d–f) The contents of TNF-*α*, IL-6, and IL-8 in culture supernatant were determined using ELISA. ^∗^*p* < 0.05 versus the control group; #*p* < 0.05 versus the IL-1*β* group.

**Figure 5:** GLA inhibits the expression of MMP-3 and MMP-13 in IL-1*β*-stimulated OA chondrocytes. Primary human OA chondrocytes were incubated with different concentrations of GLA (0, 5, 10, and 20 *μ*M) for 2 h and then stimulated with IL-1*β* (10 ng/ml) for 24 h. (a and b) The mRNA levels of MMP-3 and MMP-13 were evaluated using qRT-PCR. (c and d) The productions of MMP-3 and MMP-13 were evaluated using ELISA. ^∗^*p* < 0.05 versus the control group; #*p* < 0.05 versus the IL-1*β* group.

**Figure 6:** Modulation of ADAMTS-4 and ADAMTS-5 expression by GLA in human OA chondrocytes. Primary human OA chondrocytes were incubated with different concentrations of GLA (0, 5, 10, and 20 *μ*M) for 2 h and then stimulated with IL-1*β* (10 ng/ml) for 24 h. (a and b) The mRNA levels of ADAMTS-4 and ADAMTS-5 were evaluated using qRT-PCR. (c) The protein levels of ADAMTS-4 and ADAMTS-5 were evaluated using western blot. ^∗^*p* < 0.05 versus the control group; #*p* < 0.05 versus the IL-1*β* group.

**Figure 7:** GLA inhibited the degradation of aggrecan and collagen II induced by IL-1*β*. Primary human OA chondrocytes were incubated with different concentrations of GLA (0, 5, 10, and 20 *μ*M) for 2 h and then stimulated with IL-1*β* (10 ng/ml) for 24 h. (a and b) The mRNA levels of aggrecan and collagen II were evaluated using qRT-PCR. (c) The protein levels of aggrecan and collagen II were evaluated using western blot. ^∗^*p* < 0.05 versus the control group; #*p* < 0.05 versus the IL-1*β* group.

**Figure 8:** Modulation of NF-*κ*B signaling pathway by GLA in human OA chondrocytes. Primary human OA chondrocytes were incubated with GLA for 2 h and then stimulated with IL-1*β*. (a) The immunofluorescence was performed to assess p65 accumulation. (b and c) The levels of p-p65, p65, p-I*κ*B*α*, and I*κ*B*α* were evaluated using western blot. ^∗^*p* < 0.05 versus the control group; #*p* < 0.05 versus the IL-1*β* group.

## Data Availability

The datasets used during the present study are available from the corresponding author upon reasonable request.
